# Efficacy of Mebendazole and Praziquantel against Soil-Transmitted Helminths and *Schistosoma mansoni* Infections among Schoolchildren in Northwest Ethiopia

**DOI:** 10.1155/2021/6682418

**Published:** 2021-07-15

**Authors:** Kefale Ejigu, Tadesse Hailu, Megbaru Alemu

**Affiliations:** ^1^Amhara Public Health Institute, Bahir Dar, Ethiopia; ^2^Department of Medical Laboratory Science, College of Medicine and Health Sciences, Bahir Dar University, PO Box 79, Ethiopia

## Abstract

**Background:**

Soil-transmitted helminths (STHs) and *Schistosoma mansoni* are the main causes of morbidity among schoolchildren in the tropics. A school-based deworming program was launched to control and eliminate the infection in endemic countries including Ethiopia. Although periodic deworming is conducted in endemic areas, the prevalence of the infection is high in the country. In addition, periodic evaluation of the efficacy of the anthelminthic drug is limited.

**Objective:**

This study is aimed at checking the efficacy of mebendazole and praziquantel with the respective STHs and *Schistosoma mansoni* parasites.

**Methods:**

A longitudinal study was conducted from February to March 2018 among 422 schoolchildren. Stool samples were collected at baseline and at 2 and 4 weeks posttreatment and were processed using the Kato-Katz technique. Schoolchildren positive for STHs were treated with mebendazole and those positive for *Schistosoma mansoni* with praziquantel. After two weeks, a second round of stool was collected and examined, and then, single-dose redosing was given to each positive child. Lastly, the third stool sample was collected two weeks after the initiation of the redosing and checked for STHs and *S. mansoni* parasites. A close follow-up of students who were treated was done. All the data were entered and analyzed using SPSS version 20 for analysis. Descriptive statistics was used to compute the cure rate and egg reduction rate of mebendazole and praziquantel.

**Results:**

Among 422 participants, the prevalence of STHs, hookworm, *Ascaris lumbricoides*, and *S. mansoni* was 44.7%, 35.1%, 21.1%, and 13.9%, respectively. The cure rate of mebendazole against *A. lumbricoides* increased from 60% in the single dose to 100% in redosing after two weeks. The cure rate of mebendazole against hookworm also increased from 32.4% in the single dose to 91.0% in the redosing. The cure rate of praziquantel against *S. mansoni*-infected children was 91.5% in the first round and 100% in the redosing phase. There was a 98.6-100% egg reduction rate in the redosing regimen of both drugs.

**Conclusion:**

The cure and egg reduction rates of single-dose mebendazole in the treatment of hookworm and *A. lumbricoides* are lower at week two than at redosing, while cure and egg reduction rates of single-dose praziquantel are satisfactory to treat *S. mansoni*. Therefore, single-dose praziquantel to *S. mansoni* and redosing of single-dose mebendazole to *A. lumbricoides* and hookworm infections can be used for treatment purposes.

## 1. Introduction

Soil-transmitted helminthiasis and schistosomiasis are among the most common parasitic diseases of the neglected tropical diseases (NTDs) worldwide. Soil-transmitted helminths comprise four species of intestinal helminths, *A. lumbricoides*, *T. trichiura*, and hookworm (*Ancylostoma duodenale* and *Necator americanus*) [1, 2]. Global estimates indicated that 819 million, 439 million, and 465 million people are infected with *A. lumbricoides*, hookworm spp., and *T. trichiura*, respectively. Similarly, more than 200 million people are estimated to be infected with *S. mansoni* (WHO, 2017). In Ethiopia, an estimated 116.3 million people (comprised of 37.6 million school-age children) live in STHs and Schistosoma endemic areas [3].

*A. lumbricoides* and *T. trichiura* are transmitted via ingestion of contaminated food and/or soil whereas hookworm infection is acquired via the active penetration of the skin by the larvae. *S. mansoni* is also transmitted through skin penetration of cercaria [4]. School-age children (SAC) and preschool-age children (PSAC) are the most vulnerable population groups both for STHs and *S. mansoni* since they are playing in soil and water [5].

Heavy STH infection has a great effect on nutritional and cognitive status especially in schoolchildren due to the increased metabolic rate, anorexia, and diarrhea. These helminths also cause decreased intake or a functional increase in the body's nutrient requirement by their interference with absorptive surfaces, physical obstruction of intestinal lumen, production of proteolytic substances, and consumption of nutrients intended for the body [6, 7]. *S. mansoni* on the other hand can cause a wide range of clinical conditions that range from mild cutaneous and pulmonary manifestations to life-threatening conditions like hepatosplenic inflammation and liver fibrosis [8, 9].

The three main measures to control soil-transmitted helminthiasis and schistosomiasis include mass drug administration (MDA); water, sanitation, and hygiene (WASH); and health education. Periodic deworming of the high-risk population ensures that the levels of infection are kept below the intensity that is associated with morbidity. In Ethiopia, mebendazole (single 500 mg/kg oral dose) and praziquantel (single 40 mg/kg oral dose) are currently used in deworming programs targeting STHs and *S. mansoni*, respectively [10]. However, some livestock and human studies indicated reduced efficacy of single-dose anthelminthic therapy [11–14]. The reduced efficacy of anthelminthic drugs might be due to repeated reinfection in the endemic areas, high-intensity infection, repeated use of the same drug, and single-dose administration of anthelminthic drugs [15].

In the study area, institution-based information showed that the prevalence of STHs and *S. mansoni* infections is high though MDA is regularly given. Therefore, the aim of this study was to check the efficacy of single-dose mebendazole and praziquantel against the respective STHs and *S. mansoni* infections at day 14 and efficacy of redosing mebendazole and praziquantel against STHs and *S. mansoni* infections, respectively, after day 28.

## 2. Materials and Methods

### 2.1. Study Design, Area, and Period

A school-based longitudinal study was carried out in Andasa primary school, Bahir Dar Zuria district, Amhara region, northwest Ethiopia, from February to March 2018. The study area is located 560 km northwest of the country's capital, Addis Ababa. The elevation of the area ranges from 1700 to 2300 m above sea level. The area receives an average annual rainfall of about 1035 mm. The minimum and maximum temperatures lie at 10°C and 32°C, respectively. There are two rivers (Abay and Andasa), and people frequently encounter water contact while swimming, bathing, and washing clothes and in microirrigations. Deworming has been conducted once a year as part of a control program of STHs and *S. mansoni* infections (Figure 1).

All schoolchildren in the age range 7-18 years enrolled during the data collection time and their parents who consented and provided assent were included in the study. All schoolchildren who had taken any anthelminthic within 3 months prior to data collection were excluded. Participants were selected by systematic random sampling technique, and a total of 422 schoolchildren were included in the study.

### 2.2. Data Collection

Approximately two grams of stool was collected from each study participant using a clean, dry, and leak-proof container and applicator stick. Stool samples were transported to Amhara Public Health Institute (APHI) for laboratory processing using a cold chain. Kato-Katz thick smears were prepared and examined using a microscope by following the standard operating procedure.

In the Kato-Katz technique, feces were pressed through a mesh screen to remove large particles. A portion of the sieved stool sample was transferred through the hole of the template (41.7 mg of stool) onto a slide. After filling the hole, the template was removed and the remaining sample was covered with a piece of cellophane previously soaked in glycerol that helps to clear the fecal debris around the eggs. The Kato-Katz slides were examined with a microscope (10x followed by 40x magnification).

### 2.3. Evaluating the Efficacy of Mebendazole and Praziquantel

Training on keeping hygiene, shoe wearing, and abstinence from swimming until completing the follow-up was given for those participating schoolchildren in the study. Mebendazole (single 500 mg/kg oral dose) was provided for the children positive for *A. lumbricoides* and hookworm parasites based on the baseline results. Praziquantel (single 40 mg/kg oral dose) was also administered for schoolchildren positive for *S. mansoni*. After two weeks of initiation, a second round of single stool sample was collected and examined. And then, redosing of mebendazole (single 500 mg/kg) and praziquantel (single 40 mg/kg) oral dose was provided for those children who were positive in the second round of stool examination. A close follow-up of students to check the adverse drug reaction was done from day one to day 28. And finally, a third round of single stool sample was collected and examined two weeks after the redosing regimen.

Cure is defined as the absence of *A. lumbricoides*, hookworm, and *S. mansoni* ova or the absence of ova in the stool at day 28 of treatment. “Failure” is defined as the presence of ova of the above parasites at 28 days of treatment initiation:

(1) $$\begin{array}{c} \text{Cure rate }\left(\text{CR}\right)=\frac{\text{The number of study subjects who were negative after treatment on day }28}{\text{The total number of positive participants at baseline}}. \end{array}$$

*Egg reduction rate (ERR)*: it was calculated as the ratio of the arithmetic mean of egg count at baseline minus the arithmetic mean of egg count at follow-up divided by arithmetic mean of egg count at baseline and multiplied by 100. The efficacy of the anthelminthics was interpreted as satisfactory, doubtful, or reduced based on the reference values of the egg reduction rate [15].

### 2.4. Quality Assurance

The data quality was assured during the preanalytical, analytical, and postanalytical phases. To avoid observer bias, one slide was examined by two laboratory professionals independently. Two Kato-Katz slide smears were examined for a single participant in the second and third rounds of examination, and 15% of the Kato-Katz slides were randomly selected and checked by the principal investigator.

### 2.5. Data Entry and Analysis

All the data were entered and analyzed using Statistical Package for the Social Sciences (SPSS) version 20 software. The prevalence of *A. lumbricoides*, hookworm, and *S. mansoni* was calculated by descriptive statistics. The CR and ERR of mebendazole against *A. lumbricoides*, hookworm, and praziquantel against *S. mansoni* were computed at day 14 and day 28 of treatment by using the arithmetic mean egg count.

## 3. Results

### 3.1. Demographic Characteristics of the Study Participants

A total of 422 schoolchildren were recruited in this study. Of the total, the number of female and male participants accounted for 51.9% and 48.1%, respectively. The mean (±sd) age of the children was 11.87 (±1.98). The majority (63.5%) of the participants were in the 11-14 years age group (Table 1).

The overall prevalence of helminths and STH infection was 51.2% and 44.7%, respectively. Children in the 11-14 age group harboured the majority (33.6%) of the helminth infection. More males (28%) than females (23.2%) were infected with helminths but not statistically significant (Table 1).

The prevalence of hookworm spp., *A. lumbricoides*, and *S. mansoni* was 148 (35.1%), 89 (21.1%), and 59 (13.9%), respectively (Table 2). *Enterobius vermicularis* 4 (0.94%)*, H. nana* 2 (0.47%), and Taenia spp 2 (0.47%) were also identified. The prevalence of single, double, and triple infection accounted for 71 (32.8%), 133 (61.6%), and 12 (5.6%), respectively. Majority of the double infection was due to coinfection of hookworm and *A. lumbricoides* (22.2%). Triple infection (hookworm+*A. lumbricoides*+*S. mansoni*) *of* 5.6% was also found.

### 3.2. The Mean Egg Count and Infection Intensity of STHs and *Schistosoma mansoni*

The mean egg count for individuals with detectable eggs of *S*. *mansoni*, *A. lumbricoides*, and hookworm at the baseline fecal examination was 42, 129, and 281 eggs per gram of feces, respectively (Table 3). All *A. lumbricoides* and *S. mansoni* infections were light, and only 5.4% of hookworm infections had moderate intensity.

### 3.3. Cure Rate of Mebendazole and Praziquantel

A total of 89 schoolchildren were found to be infected with *A. lumbricoides*, and 85 of them had taken mebendazole treatment and completed the study. Among 148 hookworm-infected schoolchildren, 145 took mebendazole treatment and completed the follow-up. All 59 *S. mansoni*-infected schoolchildren took praziquantel and completed the study. We were unable to collect the 2^nd^ stool sample (at day 14) from four *A. lumbricoides-* and three hookworm-infected schoolchildren since they were absent from school.

The CR of single-dose mebendazole against hookworms and *A. lumbricoides* was 32.4% and 59.6%, respectively. Following the redosing regimen, CR of mebendazole increased to 91.0% and 100% to the respective hookworm and *A. lumbricoides*-infected children. The CR of praziquantel against *S. mansoni* in its single dose and redosing after two weeks was 91.5% and 100%, respectively (Table 4).

### 3.4. Egg Reduction Rate of Mebendazole and Praziquantel

The ERR of single-dose mebendazole against hookworm and *A. lumbricoides* infection was 53.1% and 76.4%, respectively. The ERR of mebendazole after the redosing regimen was 100% and 98.6% to the respective *A. lumbricoides* and hookworm infections. The ERR of praziquantel against *S. mansoni* in its single dose and redosing regimen was 95.1% and 100%, respectively (Table 5).

## 4. Discussion

Periodic evaluation of anthelminthic drug efficacy is ideal to overcome the burden of helminthic infections. In the present study, the prevalence of intestinal helminths at 95% CI was 51.2% (46.4-55.9%). This result is lower than the previous studies conducted in rural Bahir Dar (58%) [16] and Zarima town 82.4% [17]. This result is also comparable with the previous (54.9%) prevalence report in Durbetie town [18] but higher than a report in Libo-Kemkem (27.9%) [19] and (16.7%) in Gondar town [20]. The difference could be justified as the difference in the proper implementation of pure water, sanitation, and hygiene (WASH) and open defecation practices.

The prevalence of *A. lumbricoides* in the present study was 21.1% which is in line with a study done in Zarima town (22%) [17]. However, the present finding is higher than reports in rural Bahir Dar (1.7%) [16], Durbetie town (13.9%) [18], and Libo-Kemkem (9%) in Gondar town [20]. This could be justified as the variation in sanitation and proper utilization of latrine and endemicity of the parasite. A. lumbricoides is prevalent in areas with high altitudes.

In the present study, the prevalence of hookworm was 35.1%. This finding is higher than the previous studies conducted in Zarima town (19%) [17] and Libo-Kemkem (8.2%) [19], but lower than in rural Bahir Dar (41.3%) [16], Durbetie town (46.9%) [18], and Ethiopia (7.6%) [21]. This prevalence difference might be due to the difference in open defecation practices and shoe-wearing habits among children, the soil type, atmospheric moisture, and land surface temperature that are determinants of hookworm transmission [4].

In the present study, the prevalence of *S. mansoni* was 13.9% which is in line with previous prevalence reports in rural Bahir Dar (12.2%) [16] and in Chuahit (11.2%) [22], but lower than prevalence reports (74.9%) in Wondo Genet [23], Wolaita zone (81.3%) [24], Southern Tigray (73.9%) [25], Sanja town (35%) [26], and northwest Ethiopia (83.3%) [27]. The difference might be justified as the variation in the availability of water bodies and water contact habits of children. Children might be infected by cercaria when they are swimming, bathing, and washing their clothes in the river which is already infested with cercaria.

In the current study, the CR and ERR of single-dose mebendazole against *A. lumbricoides* were 60% and 76.4%, respectively. The current result is lower than previous study reports in northwest Ethiopia [28] and Zanzibar [29]. This could be justified as the prolonged administration of mebendazole and repeated exposure with the same type of drug in the same area can result in reduced efficacy of mebendazole.

In the present study, the CR and ERR of MEB against hookworm in single-dose treatment were 32.4% and 55.1%, respectively. Similarly, lower CR and ERR are also obtained in northwest Ethiopia [28] and in Vietnam [30]. This might be partially explained by hookworm losing its sensitivity to MEB that was previously sensitive due to the presence of alleles coding for resistance in hookworm as a result of mutations.

In the current study, the CR and ERR of MEB against hookworm and *A. lumbricoides* in redosing single-dose treatment regimen were higher than that of the single-dose regimen. This finding is consistent with a study done in northwest Ethiopia [31], Cameroon [11], and Lao PDR [32]. Since MEB is not effective in killing the eggs of *A. lumbricoides* and larvae of hookworm which become an adult within a few days, redosing gives a chance to kill these parasites.

This could be justified as redosing of MEB increases the serum half-life of the drug and is able to kill the tissue stages of the parasite in the primary dose.

The CR and ERR of single-dose praziquantel were 91.5% in the present study. This finding is comparable with a previous report [27], but higher than earlier reports [33]. The difference in the low CR and ERR might be justified as the prolonged administration of praziquantel in endemic areas.

In the present study, the CR and ERR of single-dose praziquantel treatment against *S. mansoni* were increased in the redosing regimen. This result is consistent with previous reports from northern Ethiopia [34], western Ethiopia [35], and Sudan [36]. However, the current result is higher than that of a study conducted in southern Ethiopia [23] and Niger [37]. The CR and ERR of praziquantel difference in different settings could be due to the difference in baseline infection intensity, duration of posttreatment to recheck, presence of immature stages of the parasite in the tissue, immune status, and brand of praziquantel used for treatment.

## 5. Conclusions

The single-dose regimen of mebendazole for the treatment of hookworm and *A. lumbricoides* infections showed poor cure and egg reduction rates, while redosing showed satisfactory. Single-dose and redosing regimens of praziquantel for treatment of *S. mansoni* showed satisfactory cure and egg reduction rates. Therefore, single-dose praziquantel can be used as a treatment of *S. mansoni* infection whereas single-dose mebendazole for the treatment of *A. lumbricoides* and hookworm infections should be replaced by a redosing regimen.

## Figures and Tables

**Figure 1:** Map of the study area.

**Table 1:** Demographic characteristics of the study participants with their intestinal helminthic infection status in Andasa primary school, northwest Ethiopia, 2018.

Variable		Positive, *n* (%)	Negative, *n* (%)	Total, *n* (%)
Age	7-10	58 (13.8%)	39 (9.2%)	97 (23%)
	11-14	142 (33.6%)	126 (29.9%)	268 (63.5%)
	15-18	16 (3.8%)	41 (9.7%)	57 (13.5%)

Sex	Male	118 (28%)	85 (20.1%)	203 (48.1%)
	Female	98 (23.2%)	121 (28.7%)	219 (51.9%)

Total		216 (51.2)	206 (48.8)	422 (100)

**Table 2:** Prevalence of STHs and *S. mansoni* infections among children at Andasa primary school in Bahir Dar Zuria district, northwest Ethiopia, 2018.

Helminths species	Age			Sex		Total (*n*, %)
	7-10 (*n*, %)	11-14 (*n*, %)	15-18 (*n*, %)	Male (*n*, %)	Female (*n*, %)	
*A. lumbricoides*	23 (5.45)	46 (10.9)	20 (4.7)	43 (10)	46 (10.9)	89 (21.1)
Hookworm spp	40 (9.47)	83 (19.66)	25 (5.9)	79 (18.7)	69 (16.4)	148 (35.1)
*S. mansoni*	16 (3.79)	33 (7.8)	10 (2.36)	35 (8.3)	24 (5.7)	59 (13.9)
Total	79 (18.72)	162 (38.38)	55 (13.03)	157 (37.2)	139 (32.9)	296 (70.1)

**Table 3:** Arithmetic mean of fecal egg count at baseline, after single-dose and redosing treatment of mebendazole and praziquantel among infected children in northwest Ethiopia, 2018.

Helminth species	Mean egg count per gram of stool				
	Baseline	After single dose of MEB (*N*)	After redosing of MEB (*N*)	After single dose of PZQ (*N*)	After redosing of PZQ (*N*)
*A. lumbricoides*	129	79	0	NA	NA
Hookworms	281	215	39	NA	NA
*S. mansoni*	42	NA	NA	24	0

^∗^NA = not applicable; MEB = mebendazole; PZQ = praziquantel.

**Table 4:** Cure rate of mebendazole and praziquantel among helminth-infected children of Andasa primary school in northwest Ethiopia, 2018.

Helminth spp	NIC (*N*)	NCCS (*N*)	CR of MEB (500 mg)		CR of PZQ (40 mg/kg)	
			Initial dose (*N*, %)	Redosing (*N*, %)	Initial dose (*N*, %)	Redosing (*N*, %)
*A. lumbricoides*	89	85	51 (60)	85 (100)	NA	NA
Hookworms	148	145	47 (32.4)	132 (91.0)	NA	NA
*S. mansoni*	59	59	NA	NA	54 (91.5)	59 (100)

^∗^NA = not applicable; NIC = number of infected children; NCCS = number of children who completed the study; MEB = mebendazole; PZQ = praziquantel; CR = cure rate.

**Table 5:** Egg reduction rate of mebendazole and praziquantel among helminth children of Andasa primary school in Bahir Dar Zuria district, northwest Ethiopia, 2018.

Helminth spp	NCCS	ERR of single-dose MEB		ERR of single-dose PZQ	
		Initial dose	Redosing	Initial dose	Redosing
*A. lumbricoides*	85	65 (76.4)	85 (100)	NA	NA
Hookworm spp.	145	77 (53.1)	143 (98.6)	NA	NA
*S. mansoni*	59	NA	NA	56 (94.9)	59 (100)

^∗^ERR = egg reduction rate; NA = not applicable; NCCS = number of children who completed the study; MEB = mebendazole; PZQ = praziquantel.

## Data Availability

The data used to support the findings of the study are included within the article.

## Abbreviations

STH: Soil-transmitted helminth
MEB: Mebendazole
PZQ: Praziquantel
ERR: Egg reduction rate
MDA: Mass drug administration.
